RETRACTED

# Leptin Induces Cyclin D1 Expression and Proliferation of Human Nucleus Pulposus Cells via JAK/STAT, PI3K/Akt and MEK/ERK Pathways

**DOI:** 10.1371/journal.pone.0053176

**Published:** 2012-12-31

**Authors:** Zheng Li, Jianxiong Shen, William Ka Kei Wu, Xin Yu, Jinqian Liang, Guixing Qiu, Jiaming Liu

**Affiliations:** 1 Department of Orthopaedic Surgery, Peking Union Medical College Hospital, Peking Union Medical College, Beijing, China; 2 Department of Medicine and Therapeutics, Institute of Digestive Diseases, LKS Institute of Health Science, The Chinese University of Hong Kong, Hong Kong, China; Leibniz Institute for Age Research - Fritz Lipmann Institute (FLI), Germany

## Abstract

Increasing evidence suggests that obesity and aberrant proliferation of nucleus pulposus (NP) cells are associated with intervertebral disc degeneration. Leptin, a hormone with increased circulating level in obesity, has been shown to stimulate cell proliferation in a tissue-dependent manner. Nevertheless, the effect of leptin on the proliferation of human NP cells has not yet been demonstrated. Here, we show that leptin induced the proliferation of primary cultured human NP cells, which expressed the leptin receptors OBRa and OBRb. Induction of NP cell proliferation was confirmed by CCK8 assay and immunocytochemistry and Real-time PCR for PCNA and Ki-67. Mechanistically, leptin induced the phosphorylation of STAT3, Akt and ERK1/2 accompanied by the upregulation of cyclin D1. Pharmacological inhibition of JAK/STAT3, PI3K/Akt or MEK/ERK signaling by AG490, Wortmannin or U0126, respectively, reduced leptin-induced cyclin D1 expression and NP cell proliferation. These experiments also revealed an intricate crosstalk among these signaling pathways in mediating the action of leptin. Taken together, we show that leptin induces human NP cell cyclin D1 expression and proliferation via activation of JAK/STAT3, PI3K/Akt or MEK/ERK signaling. Our findings may provide a novel molecular mechanism that explains the association between obesity and intervertebral disc degeneration.

## Introduction

The high morbidity of low back pain causes severe incapacity that increases medical expense and impacts the workforce, posing high socioeconomic costs [1]. Effective treatment of low back pain is therefore a matter of great public concern. Athough the etiology of low back pain is multifactorial, intervertebral disc degeneration (IVD) is thought to be a major cause [2]. IVD is a process that is influenced by genetic predisposition, lifestyles (e.g. occupation, smoking, alcohol consumption), co-morbidities (e.g. obesity and diabetes), and aging [3]. Several biomechanical parameters, such as height, fluid pressurization, dissipation, stiffness, and flexibility, are implicated in the initiation and progression of IVD [4]. Other factors, such as formation of cell cluster and the proliferation of fibrocartilaginous tissue, may also take part in IVD [5]. Thus far, the cause of increased cell proliferation in IVD remains unclear.

RETRACTED

First described in 1994, leptin (the 16 kDa product of the *OB* gene) is a peptide hormone secreted mainly by adipose tissues [6]. It is also produced by a variety of cells including placental cells and gastric epithelial cells [7]. Fibrocartilaginous tissues, including articular cartilage and intervertebral disc, hace been recently recognized as other sources of leptin [8]. Serum leptin levels are positively associated with body weight, implicating the involvement of this hormone in the regulation of food intake [9]. In addition, leptin is implicated in the modulation of other physiological processes, such as angiogenesis, wound healing, central and peripheral endocrine actions, and renal and pulmonary functions [10]. Emerging evidence suggest that leptin may function as a growth factor to stimulate cell proliferation in a tissue-dependent manner [11]. For instance, exogenous leptin induces sustained proliferative responses in prostate and lung eptithelial cells, pancreatic beta cells as well as breast and gastric cancer cells [12]. A recent study has shown that human herniated disc tissues and rat NP cells express leptin and its functional receptor [13]. Leptin also stimulates the proliferation of rat NP cells *in vitro* [14]. Nevertheless, it remains unclear whether leptin can induce human NP cell proliferation. Moreover, the mechanism of leptin-induced NP cell proliferation has not yet been elucidated in human or animals.

Leptin exerts its action through its cell membrane receptor that belongs to class I cytokine receptor family. Thus far, six receptor isoforms, designed as OBRa to OBRf, have been identified [15]. However, only OBRb (the long isoform of the OBR) contains intracellular motifs required for the initiation of intracellular signaling [16]. OBRb mediates the action of leptin via multiple signaling pathways, including Janus kinase/signal transducers and activators of transcription (JAK/STAT), mitogen-activated protein kinases (MAPK), protein kinase C (PKC), nitric oxide (NO), and cyclic AMP pathways [17]. In other cell types, leptin also activates extracellular signal-regulated kinase 1/2 (ERK1/2) and phosphatidylinositol 3-kinase (PI3K) in a SHP-2- and IRS-dependent manner, respectively [18]. The complexity of leptin signaling is increased by the crosstalk among these signaling pathways. The involvement of these pathways in leptin signaling in NP cells remains unknown.

RETRACTED

Obesity is an established risk factor for IVD in which leptin may play a significant role in its pathogenesis. In the present study, we determined the effect of leptin on the proliferation of primary cultured human NP cells and delineated the underlying molecular mechanism.

## Results

### Morphology, Immunofluorescence Characterization and Real-time Quantitative PCR Validation of Primary Cultured Human NP cells

After approximately 1 week, the primary cultured human NP cells reached almost complete confluence. The cells were polygonal, with multiple cytoplasmic processes and granular cytoplasm (Fig. 1A). Immunofluorescence for collagenase type II and cytokeratin 19 was observed in these cells. Figure 1C and 1D shows a typical field observed in these cultures. CA12, which was recently decribed by Minogue et al as a marker gene for human NP cells, was found to have significantly higher levels of expression in NP cells and NP tissue than in AF tissue and chondrocytes (Fig. 1D). IBSP and FBN1, which were also recently decribed by Minogue et al as negative markers gene for human NP cells, was found to have significantly low levels of expression in NP cells and NP tissue than in AF tissue and chondrocytes (Fig. 1E and 1F).

**Figure 1:** Morphology, immunofluorescence characterization and real-time quantitative PCR validation of primary cultured human NP cells. (**A**) Phase-contrast photomicrograph of primary NP cells cultured in vitro for about 1 week, just before reaching complete confluence. Original magnification, ×40. (**B**) Real-time RT-PCR analysis of novel NP cell marker gene CA12 in NP cells, chondrocytes, NP and AF. Real-time RT-PCR analysis was performed in triplicate and the expression levels of CA12 mRNAs were normalized to GAPDH mRNAs. Error bars represent standard deviration. (**C**) Fluorescence microscopy images showing collagenase type II were observed in NP cells. Nuclei were stained with DAPI, shown in blue. Images were acquired using laser scanning confocal microscopy under a 40× objective. (**D**) Fluorescence microscopy images showing cytokeratin 19 were observed in NP cells. Nuclei were stained with DAPI, shown in blue. Images were acquired using laser scanning confocal microscopy under a 40× objective. Real-time RT-PCR analysis of novel negative NP cell marker gene IBSP (E) and FBN1 (F) in NP cells, chondrocytes, NP and AF. Real-time RT-PCR analysis was performed in triplicate and the expression levels of IBSP and FBN1 mRNAs were normalized to GAPDH mRNAs.

### Human NP cells Expressed Leptin Receptors

The expression of two isoforms of leptin receptors, namely OBRa and OBRb, was determined in primary cultured human NP cells by RT-PCR and Real-time RT-PCR. Results indicated that the mRNA expression of both isoforms was detected in human NP cells (Fig. 2A and 2B), hinting at the possibility that NP cells are capable of receiving leptin signals, at least in part, via these two OBRs.

RETRACTED

**Figure 2:** Leptin stimulates NP cells growth. (**A**) The mRNA expression of OBRa and OBRb were detected in human NP cell with RT-PCR. The amplified cDNA fragments, 116 bp GAPDH, 609 bp OBRb, and 200 bp OBRa, together with DNA marker were electrophoresed. (**B**) Real-time RT-PCR analysis of OBRa and OBRb mRNA in NP cells. Real-time RT-PCR analysis was performed in triplicate and the expression levels of OBRa and OBRb mRNAs were normalized to GAPDH mRNAs. Error bars represent standard deviration. (**C**) For the dose-development studies NP cells were treated with either complete culture medium only or varying concentrations of leptin (1–1500 ng/ml) for 48 or 72 h. (**D**) For the time-development studies, NP cells were treated either complete culture medium only or leptin (10 ng/ml) for varying time intervals (24–96 h). (**E**) To further compare the cell viabilities before and after leptin treatment, NP cells were serum starved before treatment (day -1), and 1 day later treated with 10 ng/ml leptin, serum in serum-free media or vehicle (control group) over 2 days. Values are presented as mean ±SD (n = 4). The statistically differences compared with the control are noted as *p<0.05, and ***p<0.001. Data represent three independent experiments.

### Leptin Induced Human NP cell Proliferation

In serum-replete conditions, increasing concentrations of leptin (1–1500 ng/ml) significantly increased NP cell proliferation in a dose-dependent manner, with the maximal response at 1000 ng/ml at 48 h (Fig. 2C). Time-dependent induction of NP cell proliferation by leptin (10 ng/ml), a concentration within the range of plasma concentrations found in obese individuals, was observed with the maximal response at 96 h (Fig. 2D). The pro-survival effect of leptin on the loss of NP cell viability induced by serum deprivation was also examined. In this set of experiments, NP cells were pre-incubated in serum-free medium for 1 day before leptin stimulation in which serum deprivation was continuously maintained. As shown in Figure 2E, serum deprivation reduced the number of viable NP cells in all groups. Nevertheless, the number of viable cells in the leptin-treated group was signifiantly higher than that of the serum-free group but was not significantly different from the serum-replete group. This finding suggests that, in addition to its proliferative effect, leptin may maintain NP cell survival in face of nutrient starvation. The proliferative effect of leptin was confirmed immunohistochemical staining of PCNA and Ki-67 in NP cells treated with or without leptin (Fig. 3A, 3B). As shown in Figure 3C, 3F, there was a significant increase in the percentage of PCNA-positive and Ki-67-positive NP cells in the group treated with 10 ng/ml leptin as compared with the control group. Treatment with leptin (10 ng/ml) significantly increased PCNA and Ki-67 mRNA level in a time-dependent manner, with a maximal response at 48 h or 24 h respectively (Fig. 3D, 3G).

RETRACTED

**Figure 3:** Immunohistochemical staining of NP cells against PCNA and Ki-67. After 1-day serum deprivation, NP cell were treated vehicle (control), 10 ng/ml leptin in serum-free medium for 48 h. Immunohistochemical staining of NP cells against PCNA (A) and Ki-67(B). Nuclei were stained with DAPI, shown in blue. Images were acquired using laser scanning confocal microscopy under a 40× objective. PCNA-positive (C) and Ki-67(D) percentages in cultured NP cells 48 h after different concentrations of leptin and vehicle (control). Values are presented as mean ±SD. As compared with control, **p<0.01. (C–D) Real-time RT-PCR analysis of PCNA and Ki-67 mRNA expression in NP cells following leptin treatment for 0, 12, 24, 48 h, or 72 h. Real-time RT-PCR analysis was performed in triplicate and the expression levels of PCNA and Ki-67 mRNAs were normalized to GAPDH mRNAs. Error bars represent standard deviration. (E–F) NP cells were serum starved for 24 h, and then treated with vehicle (−), 10 ng/ml leptin (+), 10 µM U0126 (U0), 40 µM AG490 (AG) or 250 nM wortmannin (Wort) for 48 h. PCNA and Ki-67 mRNA expression were detected with Real-time RT-PCR analysis using GAPDH as an internal control. Error bars represent standard deviration.

### Leptin Induced STAT3, Akt and ERK Phosphorylation in Human NP cells

Leptin has been shown to instigate intracellular signaling via activation of JAK2/STAT3, PI3K/Akt, and MEK/ERK pathways in other cell types. In the present study, the effect of leptin on the activities of these pathways in human NP cells was determined by Western blot for total and phosphorylated STAT3, Akt, and ERK1/2. As shown in Figure 4, leptin stimulation time-dependently increased the phosphorylation of STAT3, Akt and ERK1/2 without altering the total protein levels. The induction of STAT3, Akt and ERK1/2 phosphorylation could be observed as early as 5 min after leptin stimulation and the maximal stimulation occurred at 30 min, 15 min and 5 min post-stimulation, respectively. These findings indicate that leptin could readily activate JAK2/STAT3, PI3K/Akt, and MEK/ERK pathways in human NP cells.

RETRACTED

**Figure 4:** Leptin activates phosphoryolations of STAT3, Akt, and ERK1/2 in NP cells. After 1-day serum deprivation, leptin (10 ng/ml) was added into the serum-free medium of NP cells for 5 min, 15 min and 30 min, and then the protein amouts of phosphorylated forms of Akt (p- Akt) (**A**), ERK1/2 (p- ERK1/2) (**B**) or STAT3 (p- STAT3) (**C**) were detected with western blotting analysis. GAPDH was also detected for a loading control.

### Pharmacological Inhibition of JAK2/STAT3, PI3K/Akt, and MEK/ERK Pathways Prevented Leptin-induced NP cells Proliferation

To examine the possible involvements of JAK2/STAT3, PI3K/Akt, and MEK/ERK pathways in leptin-induced NP cell proliferation, NP cells were treated with or without AG490 (JAK inhibitor), wortmannin (PI3K inhibitor) or U0126 (MEK inhibitor), alone or in combination, in the absence or presence of leptin. Results from CCK8 cell proliferation assays showed that AG490 or U0126 remarkably reduced leptin-induced NP cell proliferation whereas wortmannin exerted only modest inhibition. However, co-inhibition of PI3K and MEK with wortmannin and U0126 could almost completely block the proliferative effect of leptin in NP cells as in other combined treatment groups (AG490+wortmannin, AG490+U0126, AG490+wortmannin+U0126). In contrast, these inhibitors *per se* did not significantly alter NP cell proliferation, indicating that inhibition of JAK2/STAT3, PI3K/Akt, and MEK/ERK pathways specifically blocked the proliferative effect of leptin (Fig. 5).

**Figure 5:** Pharmacological inhibitors of JAK, PI3K/Akt, and MEK/ERK1/2 prevent NP cells growth from leptin induction. After 1-day serum deprivation, NP cell were treated vehicle (control), 10 ng/ml leptin (Lep), 40 µM AG490 (AG), 250 nM wortmannin (Wort), 10 µM U0126 (U0126), or 10 ng/ml leptin together with 40 µM AG490 (Lep+AG), 250 nM wortmannin (Lep+Wort), 10 µM U0126 (Lep+U0126), 40 µM AG490 and 10 µM U0126 (Lep +U0126+ AG), 40 µM AG490 and 250 nM wortmannin (Lep+AG+Wort), 10 µM U0126 and 250 nM wortmannin (Lep+U0126+Wort), 10 µM U0126, 40 µM AG490 and 250 nM wortmannin (Lep+U0126+ Wort+AG) in serum-free medium for 48 h. Values are presented as mean ±SD (n = 4). The statistically differences compared with the control are noted as *p<0.05, and ***p<0.001. Data represent three independent experiments.

### Crosstalk Among JAK/STAT3, PI3K/Akt, and MEK/ERK Pathways in Leptin-stimulated NP cells

The data presented so far indicates that JAK/STAT3, PI3K/Akt, and MEK/ERK pathways mediated the mitogenic effect of leptin in NP cells. Whether there is crosstalk among these three signaling pathways remained unclear. Western blot analysis indicates that U0126, AG490 and wortmannin significantly reduced leptin-induced ERK1/2, STAT3 and Akt phosphorylation, respectively. Interestingly, in addition to its effect on STAT3 phosphorylation, JAK2 inhibitor AG490 also partially reduced phosphorylation of ERK1/2 but not Akt induced by leptin. In contrast, MEK inhibitor U0126 reduced phosphorylation of ERK1/2, STAT3 and Akt while PI3K inhibitor wortmannin specifically reduced Akt phosphorylation induced by leptin (Fig. 6).

RETRACTED

**Figure 6:** Crosstalk among JAK/STAT3, PI3K/Akt, and MEK/ERK pathways in leptin-stimulated NP cells. After 1-day serum deprivation and then 30-min pre-treatment of vehicle (−), 10 µM U0126 (U0126), 40 µM AG490 (G) or 250 nM wortmannin (Wort), NP cells were treated with vehicle (−) or 10 ng/ml leptin (+) in serum-free media for 30 min respectively. Following, the protein amounts of phosphorylated of Akt (p- Akt) (**A**), ERK1/2 (p- ERK1/2) (**B**) or STAT3 (p- STAT3) (**C**) were detected with western blotting analyses. The same blots were stripped and reprobed with antibodies specific for total proteins of Akt, ERK1/2, or STAT3. GAPDH was also detected for a loading control. Data represent three independent expriments.

### Leptin Induced Cyclin D1 Expression in a JAK-, PI3K-, and MEK-dependent Manner

Increased cyclin D1 expression is known to promote cell cycle progression during G_1_-S transition. Here we examined the possible involvement of cyclin D1 in leptin-induced NP cell proliferation and its relationship with the JAK/STAT3, PI3K/Akt, and MEK/ERK pathways. Western blot and Real-time RT-PCR analysis show that leptin time-dependently increase cyclin D1 protein and mRNA expression in human NP cells, with the both maximal response at 72 h. Furthermore, inhibitors of JAK (AG490), PI3K (wortmannin) or MEK (U0126) blocked leptin-induced cyclin D1 protein and mRNA expression (Fig. 7).

**Figure 7:** Leptin induces NP cells’cyclin D1 expression and pharmacological inhibitors of JAK, PI3K/Akt, and MEK/ERK1/2 prevent NP cells’cyclin D1 expression from leptin induction. (**A**) After 1-day serum deprivation, NP cells were incubated in serum-free media containing 10 ng/ml leptin for varying time intervals (12–96 h), and then the amouts of cyclin D1 protein were detected with western blotting analysis using GAPDH as an internal control. (**B**) NP cells were serum starved for 24 h, and then treated with vehicle (−), 10 ng/ml leptin (+), 10 µM U0126 (U0), 40 µM AG490 (AG) or 250 nM wortmannin (Wort) for 48 h. The amouts of cyclin D1 protein were detected with western blotting analysis using GAPDH as an internal control. (**C**) Real-time RT-PCR analysis of cyclin D1 mRNA expression in NP cells following leptin treatment for 0, 12, 24, 48 h, 72 h, or 96 h. Real-time RT-PCR analysis was performed in triplicate and the expression levels of cyclin mRNAs were normalized to GAPDH mRNAs. Error bars represent standard deviration. (D) NP cells were serum starved for 24 h, and then treated with vehicle (−), 10 ng/ml leptin (+), 10 µM U0126 (U0), 40 µM AG490 (AG) or 250 nM wortmannin (Wort) for 48 h. Cyclin D1 mRNA expression were detected with Real-time RT-PCR analysis using GAPDH as an internal control. Error bars represent standard deviration.

RETRACTED

## Discussion

Increasing epidemiological evidence has supported that obesity is closely associated with IVD [19]. The cellular and molecular mechanism of obesity-related IVD, however, remains unclear. In this respect, leptin, a hormone with increased circulating levels in obese patients, has been implicated in the pathogenesis obesity-related IVD. We first characterized NP cells by assessing the morphology, the expression of collagenase type II, cytokeratin 19, CA 21, IBSP and FBN1. The results showed that NP cells in this study possessed the above these characteristics of NP cells, which was consistent with previous research [20], [21]. In this study, we demonstrated that leptin directly stimulated proliferation of human NP cells which expressed leptin receptors OBRa and OBRb. The mitogenic effect of leptin was supported by CCK-8 assay, immunostaining for two proliferative markers PCNA and Ki-67 as well as induction of cyclin D1. In this regard, disc cell proliferation is known to be associated with IVD and is likely the cause of cluster formation. In fact, proliferating cells have been found to be defective in the synthesis of normal matrix components and thereby promoting disc degeneration. These findings suggest that increased NP cell proliferation induced by leptin may be one of the possible mechanisms underlying the detrimental influence of obesity on the development of IVD; on the other hand, the effect induced by leptin on NP cell may be fine for normal intervertebral disc.

Although leptin functions as a growth factor in various types of cells, the exact mechanism of leptin-induced cell proliferation is not fully understood. In the present study, we showed that leptin-induced NP cell proliferation was accompanied with increased phosphorylation of STAT3, Akt and ERK1/2 and upregulation of cyclin D1. Inhibition of JAK, PI3K or MEK also reduced leptin-induced cyclin D1 expression and NP cell proliferation. These findings suggest that leptin induces cyclin D1 Expression and proliferation of human NP cells via JAK/STAT, PI3K/Akt and MEK/ERK pathways. Cyclin D1 is an important mediator that controls cell cycle transition from G1-to-S-phase [22]. In this regard, leptin has been shown to induce cyclin D1 in human breast and endometrial cancer cells as well as hepatocarcinoma cells[23]–[25]. To this end, the regulation of cyclin D1 and cell proliferation by JAK/STAT, PI3K/Akt and MEK/ERK signaling has been widely reported, especially in cancer biology studies [26]. Here, we demonstrate that the concomitant activation of JAK/STAT, PI3K/Akt and MEK/ERK pathways is required for induction of cyclin D1 and cell proliferation by leptin in human NP cells. In fact, other cytokines, such as PDGF, bFGF and IGF-I have been found to stimulate the proliferation of disc cells via the ERK and Akt signaling pathways and are implicated in the development of IVD [27].

RETRACTED

Leptin acts via transmembrane receptors, which are structurally similar to the class I cytokine receptor family. Leptin receptor OBR is produced in several alternatively spliced forms designated OBRa to OBRf [15]. These OBRs are expressed in a variety of tissue including lung, kidney, liver, stomach and articular cartilage [28], [29]. Among these OBRs, OBRb is the best studied and believed to be the major signal mediator of leptin. Activation of leptin receptors has been previously shown to stimulate JAK2/STAT3 pathway, PI3K/Akt and MEK/ERK pathways in other cell types [25]. Nevertheless, only sporadic studies have attempted to delineate their crosstalk. A previous study has shown that MEK inhibition blocked the activation of PI3K/Akt induced by leptin in human papillary thyroid cancer cells [30]. In line with this finding, our data suggest that leptin-induced Akt phosphorylation was dependent on MEK activity. Another important finding emerging from this work is that there is a reciprocal regulation between JAK2/STAT3 and MEK/ERK pathways, in which U0126 (MEK inhibitor) abolished STAT3 phosphorylation while AG490 (JAK inhibitor) partially reduced ERK phosphorylation induced by leptin in human NP cells. This finding is in discrepancy with those reported by Trinko *et al.* showing that U0126 blocked leptin-induced phosphorylation of ERK1/2 but not STAT3 in the central nervous system of rats [31]. Yin *et al.* also showed that JAK inhibition but not MEK inhibition prevented the growth stimulation of breast cancer cells by leptin [32]. The mechanism underlying these discrepancies, however, warrants further investigation. One of the drawbacks of this study is the lack of age-matched non-degenerate discs as control. NP cells derived from LDD patients may not necessarily reflect the in vivo scenario. This study only evaluated the effect of leptin on LDD NP cells. The comparion of the reaction of LDD and normal NP cells to leptin stimulation should provide further information for the potential involvement of leptin in LDD development. In conclusion, the evidence presented in this work indicates that leptin stimulates proliferation of human NP cells. The mitogenic effect of leptin is mediated through upregulation of cyclin D1 via concomitant activation of JAK/STAT3, PI3K/Akt, or MEK/ERK pathways that may become potential targets for pharmacological intervention. Our data also reveal an unreported signaling crosstalk among JAK/STAT3, PI3K/Akt, or MEK/ERK pathways in mediating the action of leptin. These molecular alterations constitute a possible link between obesity and an increased risk for IVD.

RETRACTED

## Materials and Methods

### Ethics Statement

All of the experimental protocols were approved by the Clinical Research Ethics Committee of the Peking Union Medicial College Hospital. Human lumbar IVD samples obtained from patients undergoing discectomy following approval from the Clinical Research Ethics Committee of the Peking Union Medicial College Hospital and fully informed written consent of patients.

### Reagents

Inhibitors were purchased from the following sources: JAK inhibitor AG490 ((*E*)-2-Cyano-3-(3,4-dihydrophenyl)-*N*-(phenylmethyl)-2-propenamide), MEK inhibitor U0126 (1,4-diamino-2,3-dicyano-1,4-bis[2-aminophenylthio] butadiene) and PI3K inhibitor Wortmannin were purchased from Sigma. All other chemicals and reagents were purchased from Sigma unless otherwise specified.

### Isolation and Primary Culture of Human NP cells

The human NP cells were dissected from patient disc surgical specimens (8 donors, 31–40 years, and average Thompson degeneration grade 2–3). All of these NP tissues was isolated from patients underwent surgeries for disc degeneration (L4/5) and not disc herniation, and therefore contact between these tissues and cells outside of the disc, these are macrophages, endothelial cells and other immune cells, were minimal or nonexistent. No granulation tissue was present. Two cell types populate the human NP: notochordal cells and chondrocyte-like cells [33]. As the notochordal cells slowly decline in abundance and appear to be absent after 10 years of age [34], NP tissues of human adolescents and adults consist of only chondrocyte-like cells. NP cells were isolated and cultured as previously described [35], [36]. Tissues specimens were first washed thrice with PBS, NP was separated from the AF using a stereotaxic microscope, then cut into pieces (2–3 mm3), and NP cells were released from the NP tissues by incubation with 0.25 mg/ml type II collagenase for 12 h at 37°C in Dulbecco’s modified Eagle medium (DMEM; GIBCO, Grand Island, NY). After isolation, NP cells were resuspended in DMEM containing 10% FBS (GIBCO, NY, USA), 100 µg/ml streptomycin, 100U/ml penicillin and 1% L-glutamine, and then incubated at 37°C in a humidified atmosphere with 95% air and 5% CO2. The confluent cells were detached by trypsinization, seeded into 35-mm tissue culture dishes in complete culture medium (DMEM supplemented with 10% FBS, 100 µg/ml streptomycin and 100U/ml penicillin) in a 37°C, 5% CO2 environment. The medium was charged every 2 days. NP cells cultured in vitro within 10 days, the second passage was used for subsequent experiments.

RETRACTED

### Reverse Transcription (RT)-polymerase Chain Reaction (PCR) for Detection of OBRa/b

Total RNA was extracted with Trizol reagent (Invitrogen, Carlsbad, CA, USA) according to the manufactuer’s instructions. The RNA was quantified by absorbance at 260 nm. cDNA was sythesized from 2 µg of total RNA using M-MLV reverse transcriptase (Invitrogen, Carlsbad, CA, USA). Oligo (dT)_18_ was used as the RT primer for the reverse transcription of mRNAs. Briefly, 2 µg total RNA with 1 µl dNTP and 1 µM Oligo (dT)_18 _in a total volume of 8 µl were denatured at 65°C for 5 min, immediately cooled on ice, and incubated with the reverse transcriptase reaction mixture supplemented with 1U RNase inhibitor in a total volume of 20 µl at 37°C for 60 min to generate the first-stand cDNA. The reaction was terminated by incubation at 55°C for 5 min and rapidly cooled on ice. The reverse-transcribed cDNA was further PCR-amplified by specific primers in 20 µl PCR mixture (cDNA, 0.25 mM NTP, 1 µM forward and reverse primers, 0.5 U Tap) for 35 cycles. The primer sets for detection of OBR and GAPDH are listed in Table 1.

**Table 1:** Nucleotide sequences of primers used in Real-time RT-PCR.

Gene	Forword Primer	Reverse Primer	Tm (°C)	Productsize (bp)
CA12	CGTGCTCCTGCTGGTGATCT	AGTCCACTTGGAACCGTTCACT	60	70
OBRa	TTGTGCCAGTAATTATTTCCTCTT	AGTTGGCACATTGGGTTCAT	56	200
OBRb	CCAGAAACGTTTGAGCATCT	CAAAAGCACACCACTCTCTC	56	609
Cyclin D1	AAC TACCTGGACCGCTTCCT	CCACTT GAGCTTGTTCACCA	56	204
PCNA	AGTGGAGAACTTGGAAATGGAA	GAGACATGGAGTGGCTTTTGT	56	154
Ki-67	TCCTTTGGTGGGCACCTAAGACCTG	TGATGGTTGAGGTCGTTCCTTGATG	56	156
IBSP	CCAGAGGAAGCAATCACCAAA	GCACAGGCCATTCCCAAA	60	68
FBLN1	CCTTCGAGTGCCCTGAGAACTA	ACCGATGGCCTCATGCA	60	74
GAPDH	TCAACGACCACTTTGTCAAGCTCAGCT	GGTGGTCCAGGGGTCTTAC	56	116

### Real-time PCR

Total mRNA was extracted from cells by using TRIzol reagent (Invitrogen, CA, USA) according to the manufacturer’s instructions. RNA was isolated with chloroform and isopropanol, washed with ethanol, and dissolved in water. Quantification of RNA was based on spectrophotometric analysis at 260/280 nm with values between 1.8 and 2.0 confirmed the purity of the RNA samples. A 2-µg sample of total RNA was reverse-transcribed with 200 U of MMLV reverse transcriptase (Invitrogen) using Oligo(dT) primers in a 20 µL reaction mixture following the manufactures’ instructions. Relative transcript levels of OBRa, OBRb, CA21, Cyclin D1, PCNA and Ki-67 mRNA were determined by real-time PCR using the iQ5 Real-Time PCR Detection System (Bio-Rad, California, USA). The real-time PCR reaction was composed of 1x SYBR Green fluorescent dye (Takara, Dalian, China), 1 µl forward primers (10 µM), 1 µl reverse primers (10 µM), 1x qPCR mix, 1 µl cDNA. The sequences of the specific primers are shown in Table. 1. To produce the melting curve, the reactions were subject to one step at 95°C for 30 s followed by 45 cycles of 95°C for 5 s, 60°C for 10 s, and 72°C for 30 s. The relative gene expression was assessed by the ΔΔCt method. GAPDH was used as an internal control.

RETRACTED

### Determination of NP cell Proliferation by Cell Counting Kit-8 (CCK8) Assay

NP cells were seeded in 96-well plates at the density of 1000 cells per well with 100 µl of complete culture medium. After adhesion for 24 hours, the medium was change to DMEM/F-12 supplemented with or without 5% (v/v) FBS and recombinant human leptin (Sigma-Aldrich, Oakville, ON, Canada) was added to the medium to final concentrations ranging from 1 ng/ml to 1000 ng/ml. The cells were then cultured for another 24, 48 or 96 h. Cells that did not exposed to leptin were used as controls and the wells to which only culture medium was added served as blanks. At the end of leptin stimulation, the supernatant was removed, and 100 µl of DMEM/F12 medium containing 10 µl of CCK8 was added to each well for another 3 h at 37°C. The culture plates were then shaken for 10 min and the optical density (OD) values were read at 450 nm.

### Immunohistochemistry for Proliferative Markers PCNA and Ki-67

Coverslips were placed into 24-well plate and then NP cells were plated and treated with or without 10 ng/ml leptin for 48 h. Afterwards, medium was removed and the cells were washed twice with PBS and fixed with 3.5% formaldehyde for 30 min at 37°C. The cells were rinsed with PBS for 3 times, permeabilized with 0.1% (v/v) Triton X-100 in PBS for 20 min and blocked with 3% (w/v) BSA and 0.05% (v/v) Tween 20 in PBS for 30 min at room temperature. After blocking, the cells were incubated overnight at 4°C with primary antibody. The antibodies used were as follows: rabbit monoclonal anti-PCNA antibody (dilution ratio 1∶500, Bioworlde, USA) and rabbit monoclonal anti-Ki-67 antibody (dilution ratio 1∶500, Bioworlde, USA). The cells were then treated with fluorescent anti-rabbit secondary antibody (1∶500, Bioworlde, USA) for 2 h at room temperature. Nuclei were stained with 4,6-diamidino-2-phenylindole (DAPI). Fluorescence images were acquired with a Leica TCS SP2 confocal microscopy (Leica, Mannheim, Germany) using the Leica Confocal Software.

RETRACTED

### Western Blot Analysis for Cyclin D1 and Total and Phosphorylated STAT3, ERK1/2 and Akt

Western blot was performed as described with modifications [37]. Briefly, total cellular proteins were extracted from NP cells with the lysis buffer and separated on 10% SDS-PAGE gel. After electrophoresis, proteins were electrotranferred onto the nitrocellulose membrane (Millipore, MA, USA). The membrane was then blocked with 5% (w/v) skim milk in TBST (20 nM Tris-HCL(pH 7.6), 137 nM NaCl, and 0.1% Tween-20), probed with appropriate primary antibodies at 4°C overnight and bound with HRP-conjugated secondary antibodies at room temperature for 1 h. Chemiluminescent signal was detected using ECL kit (Millipore, MA, USA) and autoradiography.

### Statistical Analysis

Results were expressed as means ± SD of multiple experiments. Statistical analysis was performed with Student’s t-test for comparison between two groups or an analysis of variance (ANOVA) followed by the Turkey’s *t*-test for comparison of multiple groups. *P* values less than 0.05 were considered statistically significant.
